# Skeletal Muscle-Specific CPT1 Deficiency Elevates Lipotoxic Intermediates but Preserves Insulin Sensitivity

**DOI:** 10.1155/2013/163062

**Published:** 2013-11-11

**Authors:** Wanchun Shi, Siping Hu, Wenhua Wang, Xiaohui Zhou, Wei Qiu

**Affiliations:** ^1^Department of Endocrinology, Huzhou Central Hospital, Zhejiang 313000, China; ^2^Department of Anesthesiology, Huzhou Central Hospital, Zhejiang 313000, China

## Abstract

*Objective*. By specific knockout of carnitine palmitoyl transferase 1b (CPT1b) in skeletal muscles, we explored the effect of CPT1b deficiency on lipids and insulin sensitivity. *Methods*. Mice with specific knockout of CPT1b in skeletal muscles (CPT1b M−/−) were used for the experiment group, with littermate C57BL/6 as controls (CPT1b). General and metabolic profiles were measured and compared between groups. mRNA expression and CPT1 activity were measured in skeletal muscle tissues and compared between groups. Mitochondrial fatty acid oxidation (FAO), triglycerides (TAGs), diglycerides (DAGs), and ceramides were examined in skeletal muscles in two groups. Phosphorylated AKT (pAkt) and glucose transporter 4 (Glut4) were determined with real-time polymerase chain reaction (RT-PCR). Insulin tolerance test, glucose tolerance test, and pyruvate oxidation were performed in both groups. *Results*. CPT1b M−/− model was successfully established, with impaired muscle CPT1 activity. Compared with CPT1b mice, CPT1b M−/− mice had similar food intake but lower body weight or fat mass and higher lipids but similar glucose or insulin levels. Their mitochondrial FAO of skeletal muscles was impaired. There were lipids accumulations (TAGs, DAGs, and ceramides) in skeletal muscle. However, pAkt and Glut4, insulin sensitivity, glucose tolerance, and pyruvate oxidation were preserved. *Conclusion*. Skeletal muscle-specific CPT1 deficiency elevates lipotoxic intermediates but preserves insulin sensitivity.

## 1. Introduction

Obesity and diabetes have become such big worldwide health problems. The incidences were getting higher and higher [1]. Increased intramyocellular lipid accumulation plays a very important role in obesity and diabetes, as well as their complications [2, 3]. This attracted great interest in the effect of accumulated lipid intermediates on insulin resistance [4, 5]. Lipotoxicity was regarded as the link of high levels of lipids with impaired insulin signaling [6, 7]. This sparked the interest in how excessive lipid affects *β*-oxidation and mitochondrial biogenesis, which may have a great impact on glucose utilization and insulin resistance [7–10].

Carnitine palmitoyl transferase 1 (CPT1) is an important rate-limiting enzyme of mitochondrial *β*-oxidation, by controlling the mitochondrial uptake of long-chain acyl-CoAs. Its muscle isoform, CPT1b, is the predominant isoform rich in the heart and skeletal muscles [11]. It was suggested that inhibiting CPT1 activity by specific CPT1 inhibitors alleviates insulin resistance in diet-induced obese mice [12]. However, previous studies have shown controversial results [13–15]. This brought up great concerns on the safety of this type of medications. Studies using genetic animal models may provide a better understanding. However, there is no study investigating if specific CPT1b deficiency in skeletal muscles had significant impact on lipids and insulin sensitivity.

Therefore, in this study, by establishing a mouse model, we directly explored this issue. With specific knockout of carnitine palmitoyl transferase-1b (CPT1b) in skeletal muscles of mice, we tested the following aspects: mitochondrial FAO, lipids, and insulin sensitivity.

## 2. Materials and Methods

### 2.1. Model Establishment

CPT1b M−/− mouse model was established as per previously described [12, 16, 17] by using male C57/BL6 mice (12 weeks old; 20–25 g) with Cre-lox technology [17, 18]. Mice were genotyped by standard PCR of tail DNA with PCR Master Mix (Applied Biosystems Inc.). Age-matched male littermates were used as controls (CPT1b). Twenty mice from each group (CPT1band CPT1b M−/−) were kept on a 12 h/12 h light/dark cycle, in temperature-steady rooms, and had *ad libitum* access to water and chow diet. All experimental procedures were conducted according to the Care and Use Guide of Laboratory Animals and were approved by the IAEC of the Huzhou Central Hospital.

### 2.2. General and Metabolic Profiles

General and metabolic profiles were measured at 12, 18, 24, and 30 weeks of age, including the following: body weight, lipids in serum, food intake, body mass, and fat mass, as per related protocols [19, 20].

### 2.3. RNA Extraction and Quantization

Skeletal muscle mRNA and protein were extracted and purified with standard protocols as per our previous protocols [7, 21]. RT-PCR was performed for mRNA quantization per standard protocols with the reagents from ABI system Inc. Primers were designed with Primer Express and made by Invitrogen Inc. Quantitative real-time RT-PCR analyses were carried out by using Step one real-time PCR system (Applied Biosystems Inc.). Cycles were 50°C for 2 min, a 2 min 95°C denaturing step, followed by 50 cycles of 95°C denaturation, incubated at 60°C for 2 min, and denatured at 95°C for 1 sec for the final step. Results were normalized to *β*-actin. The sequences of the primers are as follows: for CPT1b: forward: GAC CAT AGAGGC ACT TCT CAGCAT GG, reverse: GCAGCA GCTTCA GGG TTTGT; *β*-actin: forward: GTC CTC TCC CAA GTC CAC AC, reverse: GGG AGA CCA AAA GCC TTC AT; pAkt forward: TAA TAC GAC TCA CTA TAG GGC CAA GGAGATCATGC, reverse: GATTTAGGTGACACTATAGCTCCAAGCTATCGTCC; Glut4 forward: ACCGTGGTCCTTIGCTGTGTT, reverse: ACC CCA ATG TTG TAC CCA AAC T.

### 2.4. CPT1 Activity Measurement

As described previously [16, 22, 23], a modified mitochondrial CPT1 assay was performed to measure CPT1 activity. Briefly, quantified mitochondria (100 *μ*g protein) from skeletal muscles were incubated with reaction buffer (117 Mm Tris-HCl, 0.28 mM reduced glutathione, 4.4 mM ATP, 4.4 mM MgCl_2_, 16.7 mM KCl, 2.2 mM KCN, 40 mg/l rotenone, 0.1% BSA, and 50 mM palmitoylCoA) at 37°C for 5 min. Initiate the reaction by adding 2 mM [^14^C]-carnitine (0.1 *μ*Ci) and queued it 10 min later with 50 *μ*L 1.2 mM ice cold HCl. [^14^C]-palmitoyl carnitine was extracted with water saturated butanol and measured via liquid scintillation counting.

### 2.5. Fatty Acid Oxidation (FAO) Measurement

As previously described [24, 25], FAO was examined with radiolabeled palmitate FAO assay. Skeletal muscle tissues were homogenized, and mitochondria were isolated and quantified (100 *μ*g proteins). Palmitate oxidation assay was performed with reaction buffer (75.5 mM sucrose, 12.5 mM K_2_HPO_4_, 100 mM KCl, 1.75 mM MgCl_2_-6H_2_O, 1.75 mM L-carnitine, 0.125 mM L(-) malic acid, 1.75 mM DTT, 0.07 mM NAD+, 2 mM ATP, 10 Mm Tris-HCl, and 0.07 mM Coenzyme A). The reaction started when 200*μ*M [^14^C]-palmitate-15% BSA (1 : 6) complex (0.04 *μ*Ci/reaction mixture) was added and stopped by 3.5 M perchloric acid after incubation at 37°C for 30 min. CO_2_-trapping medium (NaOH, 0.1 M) for ^14^C radioactivity was measured by liquid scintillation to calculate palmitate oxidation rate. After incubation, ^14^CO_2_ and ^14^C-ASPs were measured (LS 6500; Beckman Coulter). All assays were performed in triplicate, and data were normalized to protein content. Calculations were then performed accordingly. 

### 2.6. TAGs, DAGs, and Ceramides Measurement

As previously reported [26–28], TAGs, DAGs, and ceramides were tested with KC-ESI-MS and gas chromatography (Applied Biosystems Inc.). Skeletal muscle tissue homogenates were extracted according to the protocol. Samples for ceramides were spiked with 50 ng C17:0. After the solution was evaporated dry and reconstituted, the samples were analyzed with mass spectrometry (MS). The analysis was performed in positive ion mode electrospray ion (ESI-MS) source and precursor ion scans *m*/*z* 264 and 282 (ceramides). Ceramides were quantified by taking the ratios of the integrated intensity for each subspecies to the intensity of C17:0. 

### 2.7. Insulin Tolerance Test and Glucose Intolerance Test

As described [29–31], insulin tolerance test and glucose intolerance test were performed at 31 weeks of age. An intraperitoneal glucose tolerance test (iGTT) and insulin tolerance test (ITT) were performed on nonanaesthetized mice after 8 hours' fasting. Blood glucose was measured with lancet glucometer (Johnson and Johnson). For iGTT, 20% glucose (2.0 g/kg body weight) was administered intraperitoneally. Blood samples were collected from tail vein at 30, 60, 90, and 120 min for glucose levels. For ITT, glucose blood levels were sampled at 5, 10, 15, 20, 25, and 30 min following intraperitoneal injection of human insulin (0.75 U 4.5 nmol/kg; Novolin R, Novo Nordisk). 

### 2.8. Glucose Oxidation (Pyruvate Oxidation)

As described previously [32, 33], skeletal muscles were homogenized in ice-cold buffer (250 mM sucrose, 10 mM Tris-HCl, 2 mM EDTA, and 1 mM ATP (pH 7.4)). For glucose oxidation, fresh skeletal muscle tissues were homogenized in ice-cold buffer (5 mM KCl, 2 mM Tris-HCl, 0.5 mM Tris base, 0.25 mM MgCl_2_-6H_2_O, 0.05 mM EDTA, and 0.05 mM ATP (pH 7.4)), 400 *μ*L homogenate was used and the reaction started when 200 *μ*M [^14^C]-glucose (0.1 *μ*Ci/reaction mixture) was added. The reaction buffer and condition are the same for palmitate oxidation as described above. CO_2_-trapping medium (NaOH, 0.1 M) for ^14^C radioactivity was measured by liquid scintillation to calculate glucose oxidation and quantified by weight of the skeletal muscle tissue homogenate.

### 2.9. Statistical Analysis

SAS 9.3 (SAS Institute Inc.) was used for data analysis. All data are presented as the mean ± SD. Student's *t*-test was used to evaluate the statistical significance of differences between knockout and controls. *P* < 0.05 was regarded as significant. 

## 3. Results

### 3.1. CPT1b M−/− Model with Impaired Muscle FAO

As shown in Figure 1(a), the mRNA expression of CPT1b decreased specifically in skeletal muscles (RT-PCR) but not in the heart muscle in CPT1b M−/− mice. It is barely expressed in kidney or liver regardless of knockout or not. CPT1 activity is barely detectable (DTNB assay at 412 nm) in mitochondria (Figure 1(b)) for the knockout mice, even up to 10 minutes. This indicated the successful establishment of this model. 

### 3.2. General and Metabolic Profiles

Compared to the mice in CPT1b group, those mice in CPT1b M−/− group had similar daily food intake. However, as shown in Table 1, their body weights were lower, starting about 12 weeks of age, along with lower fat mass (*P* < 0.05, resp.). Their lipids levels were higher (*P* < 0.05), but their glucose and insulin levels were similar.

### 3.3. Impaired Mitochondrial FAO and Lipid Accumulation

As shown in Figure 2(a), FAO was decreased in isolated mitochondria (radiolabeled palmitate) in skeletal muscles of CPT1b M−/− mice. This was accompanied by elevation of ceramides, TAGs, and DAGs (Figures 2(b) and 2(c)). Interestingly, for the ceramides, C16, C18, and C18:1 had significant increases for CPT1b M−/−, but not for C24 or C24:1. Both DAGs and TAGs are dramatically elevated in CPT1b M−/− mice. 

### 3.4. Preserved Insulin and Enhanced Glucose Sensitivity. 

As shown in Figure 3(a), CPT1b M−/− mice maintain insulin sensitivity (insulin tolerance test). Compared with wild type, glucose tolerance test of CPT1b M−/− mice had improved significantly (as shown in Figure 3(b)). Pyruvate oxidation went up (Figure 3(c)) and so did insulin-stimulated pAkt and GLUT4 (Figure 4). This suggested that insulin sensitivity and glucose homeostasis were improved in CPT1b M−/− mice.

## 4. Discussion

The relationship of fatty acid oxidation, lipids accumulation, and insulin sensitivity in skeletal muscles has been quite interesting. Imbalanced fatty acid uptake and fatty acid oxidation (FAO) have been linked to insulin resistance in muscles, which in turn worsens and complicates obesity and diabetes, as well as their complications [7, 34, 35]. The findings have been quite controversial. 

Some studies showed that increasing fatty acid oxidation alleviated insulin resistant [36]. Our study demonstrated that in mice with conditional knockout CPT1b in skeletal muscles, mitochondrial fatty acid oxidation was depressed dramatically. This was accompanied by increased accumulation of lipids in skeletal muscles, such as DAGs, TAGs, and ceramides. Regardless of these changes, insulin tolerance test, glucose tolerance test, and pyruvate oxidation all proved better insulin sensitivity for the knockout mice. This is partially consistent with the recent results in high-fat diet-induced obese mice, when given CPT1 inhibitor oxfenicine [10], as far as the major findings are concerned. But for the lipids accumulation, they showed that fatty acid intermediates decreased. Another study done with different CPT1 inhibitor, etomoxir, suggested that lipids intermediates increased [37]. Interestingly, this was correlated with impaired glucose disposal from skeletal muscles. Since about 70% of total insulin-induced glucose disposal occurs in skeletal muscles, this may indicate that increased fatty acid intermediates in skeletal muscles could damage insulin sensitivity. This is not the case shown in our study. On the contrary, our study showed that regardless of the characteristics of lipids accumulation, the mice are still insulin sensitive.

This is very exciting. There may be many pathways involved. First, due to the knockout of CPT1b in skeletal muscles, the major fuel sources were in deficit. This may suggest that signaling pathways related to energy were impaired or injured such as AMPK or mTOR [38]. Second, abnormal mitochondrial biogenesis and mitochondrial dysfunction may contribute to insulin resistance and diabetes [39, 40]. We explored from these aspects the enzymes involved in mitochondrial activity such as *β*-HAD and citrate synthase, genes related to transcriptions such as NRF (nuclear respiratory factor), and the major nuclear receptor activator PGC1*α* [7]. Thirdly, considering the correlation of adaptation of peroxisomal and amino acid to mitochondria, we further explored these changes. We will report these results in our next paper and further discuss the mechanism involved.

In summary, our study finding is very unique. It suggested that with specific knockout of CPT1b in skeletal muscles, although there were lipids accumulations in skeletal muscles, the insulin sensitivity still remains. This may point towards a great direction for pharmaceutical development.

## Figures and Tables

**Figure 1:** (a) CPT mRNA expression in different tissues, compared between wild type with CPT1b and knockout mice with CPT1b M−/−. It showed that the expression of CPT1b was significantly reduced in gastric and skeletal muscles (*P < 0.05). (b) CPT1 activities were reduced in knockout mice compared with wild type, significant at 2, 4, 6, 8, and 10 minutes (*P < 0.05). *n* = 20 for each group.

**Figure 2:** (a) Basal mitochondrial FAO was reduced in the skeletal muscle of knockout mice, compared with wild type (*P < 0.05). (b) Ceramides were accumulated in skeletal muscles of knockout mice, especially for C16 and C18 (*P < 0.05) but not for C18:1 or C24 or C24:1. (c) DAGs and TAGs were accumulated in skeletal muscles of knockout mice (*P < 0.05). *n* = 20 for each group.

**Figure 3:** Insulin tolerance test showed the knockout mice preserved insulin sensitivity (a) with better glucose tolerance test (b) and improved glucose metabolism (c). *n* = 20 for each group. *P < 0.05.

**Figure 4:** RT-PCR for pAkt and Glut4 showed preserved expression with CTP1b specific knockout. *n* = 20 for each group. *P < 0.05.

**Table 1:** General and metabolic profiles at 30 weeks of age.

Profiles	CPT1b	CPT1b M−/−	*P* value (CPT1b versus CPT1b M−/−)
Body weight (gram)	35.1 ± 2.2	26.3 ± 1.1	<0.05
Fat mass (gram)	15.2 ± 1.0	5.1 ± 0.4	<0.05
TAG in serum (ng/dL)	100.3 ± 2.1	150.1 ± 2.9	<0.05
DAG in serum (ng/dL)	10.3 ± 0.1	14.1 ± 0.2	<0.05
Fasting glucose (mg/dL)	105.1 ± 5.2	102.5 ± 4.3	NS
Fasting insulin (ng/mL)	2.0 ± 0.1	2.3 ± 0.1	NS
